This article has been retracted.

# Classification and Detection of Mesothelioma Cancer Using Feature Selection-Enabled Machine Learning Technique

**DOI:** 10.1155/2022/9900668

**Published:** 2022-07-27

**Authors:** M. Shobana, V. R. Balasraswathi, R. Radhika, Ahmed Kareem Oleiwi, Sushovan Chaudhury, Ajay S. Ladkat, Mohd Naved, Abdul Wahab Rahmani

**Affiliations:** ^1^SRM Institute of Science and Technology, SRM Nagar, Kattankulathur, Kanchipuram, 603203, Chennai, India; ^2^Department of Networking and Communications, School of Computing, SRM Institute of Science and Technology, Kattankulathur, India; ^3^Department of Computer Technical Engineering, The Islamic University, 54001 Najaf, Iraq; ^4^University of Engineering and Management, Kolkata, India; ^5^Department of Instrumentation Engineering, Vishwakarma Institute of Technology, Pune, India; ^6^Amity International Business School (AIBS), Amity University, Noida, India; ^7^Isteqlal Institute of Higher Education, Kabul, Afghanistan

## Abstract

Cancer of the mesothelium, sometimes referred to as malignant mesothelioma (MM), is an extremely uncommon form of the illness that almost always results in death. Chemotherapy, surgery, radiation therapy, and immunotherapy are all potential treatments for multiple myeloma; however, the majority of patients are identified with the disease at an advanced stage, at which time it is resistant to these therapies. After obtaining a diagnosis of advanced multiple myeloma, the average length of time that a person lives is one year after hearing this news. There is a substantial link between asbestos exposure and mesothelioma (MM). Using an approach that enables feature selection and machine learning, this article proposes a classification and detection method for mesothelioma cancer. The CFS correlation-based feature selection approach is first used in the feature selection process. It acts as a filter, selecting just the traits that are relevant to the categorization. The accuracy of the categorization model is improved as a direct consequence of this. After that, classification is carried out with the help of naive Bayes, fuzzy SVM, and the ID3 algorithm. Various metrics have been utilized during the process of measuring the effectiveness of machine learning strategies. It has been discovered that the choice of features has a substantial influence on the accuracy of the categorization.

## 1. Introduction

Cancer of the mesothelium, often known as malignant mesothelioma (MM), is an exceedingly rare but fatal type of the disease. It is possible to treat multiple myeloma with chemotherapy, surgery, radiation therapy, and immunotherapy; however, the majority of patients are diagnosed with the illness at an advanced stage, at which point it is resistant to these therapies. The median amount of time someone survives after receiving a diagnosis of advanced multiple myeloma is one year. Asbestos, a substance that was used extensively around the world in the 1970s and 1980s, has a significant connection to mesothelioma (MM) [1, 2].

Due to the fact that multiple myeloma cases have continued to climb despite the fact that the use of asbestos has been prohibited ever since the turn of the twenty-first century, the disease's extended latency period is to blame [3]. The most important diagnostic technique for multiple myeloma is the histological investigation, which should also be supported by clinical and radiographic findings (MM). The definite diagnosis of multiple myeloma (MM), which is required for the proper treatment of the disease, is crucial from both a medical and a legal aspect. The effective treatment of the illness is essential for survival. However, a precise diagnosis may be difficult to arrive at in the earlier stages of multiple myeloma [4, 5]. This is due to the fact that there is a great deal of variation between individual cases and traits that are shared with other malignancies or benign or reactive processes. In addition, as multiple myeloma has a very low prevalence, pathologists are often inexperienced with the illness and fail to recognize it due to this lack of familiarity [5].

CFS takes into account not only the unique ability of each characteristic but also the degree of overlap that occurs between those features in order to determine the worth of a certain collection of attributes. Examples of characteristics that are selected are those that have a high correlation with the class but a low intercorrelation with the other qualities [6].

This paper presents classification and detection of mesothelioma cancer using feature selection-enabled machine learning technique. First features are selected using CFS correlation-based feature selection method. It is a filter which selects relevant features for the classification. It results in improving the accuracy of classification model. Then, classification is performed using fuzzy SVM, naïve Bayes, and ID3 algorithm.

## 2. Literature Survey

In this article, a review of current research on feature selection, dimensionality reduction, and classification is offered. A variety of methodologies are now being used in an effort to assess cancer data in the most efficient manner feasible. It is challenging to create and assess prediction models due to the small sample size of the cancer data as well as the high complexity of the data.

According to Kar et al. [7], the adaptive *K*-Nearest Neighborhood- (KNN-) based gene selection approach and the PSO method were both suggested in order to choose just a limited group of relevant genes that are adequate for the intended classification purpose. Both of these approaches are based on the idea that the KNN is the neighborhood with the most similar genes. Chen et al. [8] presented the PSOC4.5 method, which combines PSO with C4.5-based feature selection. To test the effectiveness of this method, the researchers used 10 different datasets. You may pick from one of five subsets of the dataset that are all the same size but do not overlap with one another. During the evaluation phase, each subset is used only once, and the remaining four runs are put into the training process. After that, we proceed to get the averages from these results. The model's overall performance was evaluated based on how accurately it classified new data. The recommended method worked far better than the ones that were attempted before that were relevant to the problem at hand. When using the suggested models, using five folds and five runs resulted in an average accuracy of 97.52 percent for 11 tumors, 74 percent for 14, 74 percent for 9, and 56.34 percent for brain tumor 1, 85.75 percent for brain tumor 2, and 100 percent for leukemia. The accuracy of the leukemia prediction was 100 percent, one hundred percent in the case of lung cancer, 92.49 percent in the case of SRBCT, 94.11 percent in the case of prostate cancer, and 91.88 percent in the case of DLBCL.

Garro et al. [9] came up with the notion that the artificial bee colony (ABC) feature selection approach is superior to other methods. They asserted that they designed this model utilizing the bee's hired bees, bystanders, and scouts based on the principles of the bee's division of labor. This was based on the fact that the bee has a division of labor. In order to train the algorithm, microarray datasets relating to All-AML leukemia, breast cancer, prostate, and diffuse large B cell leukemia are used (DLBCL). The model achieved a classification accuracy of 85.6 percent after training and testing on breast cancer with 0.1 thresholds, whereas the overall accuracy of the model was 65.3 percent. When the threshold value is increased from 0.1 to 0.5, the performance of the system is shown to rise to 84.2 percent during testing; but, during training, the performance is shown to decrease to 83.3 percent.

When it comes to classifying the information contained in microarrays, Nguyen and his colleagues [10] came up with a method of selecting genes collectively. The Analytic Hierarchy Process (AHP), in its modified form, is used as the foundation for gene selection. The modified AHP may be used to handle two-sample *t*-tests, entropy tests, receiver operating characteristic curves, Wilcoxon tests, and signal-to-noise ratios, among other statistical tests and analyses (MAHP). In the process of gene selection, a singular strategy is not optimal; hence, these researchers developed a way to address the problem of individual ranking approaches. Before being included in the final analysis, the method's top-ranking genes were put through a classification process that included the usage of SVM, MLP, KNN, LDA, and PNN. They train the model using LOOCV because it works well with very few samples and is thus more efficient. When attempting to measure performance, they make use of accuracy, sensitivity, and specificity.

Sasikala et al. [11] propose employing game theory in conjunction with an optimization strategy for the purpose of feature selection for supervised classification. The Shapely Value Embedded Genetic Algorithm (SVEGA) is a novel adaptive feature selector for multiclass classification that is based on game theory and optimization techniques. Its goal is to improve detection accuracy while also selecting the best possible subset of features. In order to determine whether or not there was a difference between the selected features and the original datasets, the recommended method for selecting features was put through its paces. SVEGA was evaluated in comparison to the SVM, NB, KNN, C4.5, and ANN classifiers, which are all quite prevalent.

Moayedikia et al. [12] presented the feature selection approach called SYMON, which employs symmetric uncertainty and harmony search, in order to solve the problem of classifying large dimensions of unbalanced class datasets. This approach was developed in order to solve the problem of classifying large dimensions of unbalanced class datasets. In order to overcome the difficulty of classifying the datasets, this solution was implemented. They make use of a method that is referred to as “hold-out,” which gives them the ability to utilize samples that were not employed in the process of creating the model. Training, validation, and testing samples are the names given to the three separate subsets that make up the dataset. These subsets are referred to by their respective titles, using DNA microarrays to collect data and having eight distinct datasets. First, the cost of computation for SYMON is rather high, and second, the flexible subset properties of the method make it hard to find a solution that is optimal.

A mixture of Fuzzy Backward Feature Elimination (FBFE) and Independent Component Analysis (ICA) was utilized by Aziz et al. [13] to improve the accuracy of SVM and NB classifiers. This was accomplished by using both techniques. They combine the ICA and FBFE algorithms, both of which are extensions of the PCA, and use this combination for feature selection. After utilizing ICA to determine the most important traits beforehand, researchers then turn to FBFE and ICA to decide which genes should be included in the optimal subset.

Tabakhi et al. [14] used the Ant Colony Optimization (ACO) algorithm into the filter process in order to reduce the number of redundant genes and increase the number of genes that are relevant to the study. MGSACO is a technique of gene selection that does not involve any supervision. During the course of an iterative process for making improvements, a population of agents will choose a subset of genes at each stage of the process. The performance of the newly found subset of genes is evaluated with the use of a fitness function once this step has been completed. The final gene collection is composed of those genes that have consistently shown strong performance throughout all of the iterations. SVM, NB, and DT were the three different classifiers that were used in order to analyze and categorize the genes that were found. The error rate of their model was 1.4 for SVM, 2.0 for NB, and 1.5 for DT, respectively; the data suggest that error rate was utilized to evaluate model performance with relevant research. In the future, they suggest developing a metric for assessing the quantity of selected genes present in each individual ant, in addition to developing other fitness functions, in order to enhance the efficiency of the gene selection process.

Sreepada et al. [15] proposed for the use of a hybrid approach, which would combine filters and wrappers in order to take use of the most beneficial aspects of both approaches. The approach is put to the test using three different datasets: those pertaining to the colon, DLBCL, and leukemia, respectively.

Hesitant fuzzy sets (HFSs), as described by Ebrahimpour and Eftekhari [16], have the potential to be used as a feature selection technique for the purpose of the classification of data pertaining to cancer. They were driven to do the sequential forward search by the correlation-based feature selection (CFS). This research made use of a total of nine binary class microarray datasets, two of which were known as the Smk and Gli85 ovarian microarrays. This methodology may be broken down into a total of three stages. The first phase in the process of creating hesitant fuzzy sets is looking for qualities that are redundant with one another by using similarity measures. In the second stage, ranker algorithms are used to quantitatively assess the importance of the relationships between the various features and class labels. The third stage of the method consists of the computer doing a sequential forward search for the subset of desired qualities.

Feature detection, classification, and performance evaluation are all components of a technique that may be broken down into three distinct phases, as stated by Al-Rajab et al. [17]. The model was validated using the dataset pertaining to colon cancer. First and foremost, we investigated the criteria that are used to pick and then categorize characteristics. In the third and final phase, you will engage in introspection and analysis. Information gain (IG), particle swarm optimization (PSO), and genetic algorithm (GA) were the algorithms that were used in the feature selection process (IG). It was decided to use SVM, naive Bayes, and GP as classifiers, while the Weka tool was used as a development aid. Utilizing the particle swarm optimization (PSO) approach proved to be the most effective method. Other algorithms were unable to compete with this combination (94 percent). It is feasible that the method developed by the authors might be used to the selection and classification of cancer datasets other than colon cancer.

A method to feature selection that is based on an adaptive genetic algorithm (AGA) and mutual information maximization (MIM) was developed by Lu et al. [18]. This technique is known as MIMAGA. The proposed model was verified by employing six different microarray cancer datasets, including leukemia, colon cancer, prostate cancer, lung cancer, and breast cancer, with the exception of SRBCT, which is a four-class dataset. These datasets were used to test the model's accuracy. The proposed model was evaluated with the assistance of four distinct classifiers, including the BPNN, SVM, ELM, and Regularized Extreme Learning Machine (RELM). The results obtained using the recommended approach were evaluated and contrasted with those obtained using more conventional feature reduction techniques such as information gain and principal component analysis (PCA).

Combining Artificial Intelligence (AI) with fuzzy logic allows one to take advantage of the distinct advantages offered by both AI and ANN classification capabilities. As a result, it is possible to develop an effective and precise hybrid classifier even in situations in which there is an insufficient amount of data. Because fuzzy parameters rather than crisp parameters are used in the training process of the proposed model, it requires fewer training samples than conventional nonfuzzy neural networks. As a result, it may learn better than the conventional neural network and provide more accurate results than the conventional neural network. Models such as LDA, QDA, *K*-Nearest Neighbor, and SVM, along with other statistically intelligent techniques and typical artificial neural networks, are compared to the one that was recommended (SVM). One component of the model is not hierarchical, whereas the other component of the model is hierarchical. The model consists of two components (hierarchical). The performance of the model yields a classification error rate that is 6.3 percent and 8.3 percent for the training dataset and 3.7 percent and 4.4 percent for the testing dataset, respectively.

## 3. Methodology

This section presents classification and detection of mesothelioma cancer using feature selection-enabled machine learning technique. First, features are selected using CFS correlation-based feature selection method. It is a filter which selects relevant features for the classification. It results in improving the accuracy of classification model. Then, classification is performed using fuzzy SVM, naïve Bayes, and ID3 algorithm. The block diagram is shown in Figure 1.

CFS takes into account not only the unique ability of each characteristic but also the degree of overlap that occurs between those features in order to determine the worth of a certain collection of attributes [19]. Examples of characteristics that are selected are those that have a high correlation with the class but a low intercorrelation with the other qualities [20].

The categorizing approach may be used in either a supervised or particularly unsupervised manner, depending on the researcher's preference [21]. This is a truth that is well recognized. As a direct consequence of this, support vector networks are now considered to be machine learning standards that are being monitored. It is possible to utilize a support vector machine (SVM) to create feature points or attribute states by using nonlinear hyperplanes and planar projections [22]. The use of support vector machines is significantly influenced by the utilization of Gaussian kernels, the variance and standard deviation of the data, and the methods that were utilized to compute the kernels. You may train a machine learning model to recognize only one class at a time by using fuzzy support vector machines (fuzzy SVM). The SVM was unable to pinpoint any locations where eruptions were taking place. In this way, FSVM is being put to productive use. Data that are stochastic and probabilistic need to have prelearning data performed on them. The topic of discussion in this section is stochastic relationships.

The construction of metadata using these naïve Bayes classifiers makes use of both factual and probabilistic data. In this particular instance, the Bayes hypothesis (H) and predictions based on fundamental freedom are underlined. Since it was initially brought to light in the 1950s, a significant number of individuals have been paying attention to it ever since then. Research in the field of medical diagnostics, data on spatial imaging, and the organization of information are only some of its numerous uses [23]. This classifier contains a vast variety of customizable indicators and requires a wide variety of parameters to function properly [24].

ID3 is credited as being one of the people who first developed it. This was the very first strategy based on a decision tree that was ever developed [25]. In addition to the notion of entropy, this approach makes use of the idea of information gain. Calculating the functional characteristic entropy in an iterative manner requires us to begin with a nodule as our point of departure. In the context of entropy and information gain, split attributes are datasets that have been partitioned into subsets based on the error rate that is the lowest among them [26]. This is how the theory of split attributes proposes that split attributes should work (entropy). In the absence of a specific classification of the target classes, all the algorithm does is repeat through its own stages for each individual subset of data [27]. The nodes that are part of a branch but are not considered to be its terminal nodes are referred to as the branch's terminal nodes. The split attribute allows for the identification of nonterminal nodes in a tree, which is possible given that these nodes do in fact exist [6, 28].

## 4. Result Analysis and Discussion

Mesothelioma dataset [29] consists of 324 instances and 34 features. CFS feature selection algorithm is applied for feature selection. It selects 14 features. Then, machine learning algorithms like fuzzy SVM, naïve Bayes, and ID3 algorithm are applied to classify data. Accuracy, specificity, and sensitivity parameters are used to measure the performance of machine learning techniques for mesothelioma detection. Results are shown in Figures 2–4.

(1) $$\begin{array}{c} \text{Accuracy}=\frac{\text{TP}+\text{TN}}{\text{TP}+\text{TN}+\text{FP}+\text{FN}},\\ \text{Sensitivity}=\frac{\text{TP}}{\text{TP}+\text{FN}},\\ \text{Specificity}=\frac{\text{TN}}{\text{TN}+\text{FP}}, \end{array}$$

where

(2) $$\begin{array}{c} \text{TP}=\text{true positive},\\ \text{TN}=\text{true negative},\\ \text{FP}=\text{false positive},\\ \text{FN}=\text{false negative}. \end{array}$$

During the first phase of the feature selection process, the CFS correlation-based feature selection technique is used. It performs the function of a filter, choosing just the characteristics that are pertinent to the categorization. As a direct result of this, the accuracy of the model used for categorizing data is much increased. Following that, classification is performed with the assistance of naive Bayes, fuzzy support vector machines, and the ID3 method. During the process of determining how successful certain machine learning algorithms are, a number of different measures have been applied. It has been shown that the selection of characteristics has a significant impact on the precision of the classification process.

## 5. Conclusion

Cancer of the mesothelium, also known as malignant mesothelioma (MM), is a very rare type of the disease that nearly always ends in the patient's death. Numerous myelomas have multiple possible treatments, including chemotherapy, surgery, radiation therapy, and immunotherapy; however, the majority of patients are diagnosed with the illness at an advanced stage, when it is resistant to these therapies. One year is the typical amount of time that a person has left to live after receiving the diagnosis that they have advanced multiple myeloma after they have received this information. The risk of developing mesothelioma is significantly increased when a person has been exposed to asbestos (MM). Using an approach that enables feature selection and machine learning, this article proposes a classification and detection method for mesothelioma cancer. The CFS correlation-based feature selection approach is first used in the feature selection process. It acts as a filter, selecting just the traits that are relevant to the categorization. The accuracy of the categorization model is improved as a direct consequence of this. After that, classification is carried out with the help of naive Bayes, fuzzy SVM, and the ID3 algorithm. Various metrics have been utilized during the process of measuring the effectiveness of machine learning strategies. It has been discovered that the choice of features has a substantial influence on the accuracy of the categorization.

## Figures and Tables

**Figure 1:** Classification and detection of mesothelioma cancer using feature selection-enabled machine learning technique.

**Figure 2:** Accuracy of machine learning classifiers for mesothelioma detection.

**Figure 3:** Sensitivity of machine learning classifiers for mesothelioma detection.

**Figure 4:** Specificity of machine learning classifiers for mesothelioma detection.

## Data Availability

The data shall be made available on request.
